RETRACTED

# Dance-Specific Action Recognition Method Based on Double-Stream CNN in Complex Environment

**DOI:** 10.1155/2022/9327277

**Published:** 2022-08-30

**Authors:** Yan Jin

**Affiliations:** Shanghai Normal University Music College, Shanghai 200234, China

## Abstract

Technology for dance-specific motion recognition is widely used in many industries, but Chinese research in this area is still in its early stages. Recognizing specific dance movements is the key to learning about and comprehending human actions and behaviors. The fault-tolerant feature of standardized sign language recognition is extended under the condition of small sample sizes, but the recognition accuracy remains a challenge. This issue needs to be resolved by fusing the essential details of particular dance movements. A dual-stream convolution neural network is suggested in this paper to investigate the recognition of particular dance movements. In this paper, a dual-stream convolution neural network is used to study the recognition of particular dance movements. The time spent by this algorithm gradually increases as the number of people in the image does, but only slightly. The algorithms proposed by Bergonzoni (2017) and Liu et al. (2021) both experience linear increases in running time as the population grows. In contrast, the running time of the algorithm in this study essentially increases negligibly. It has become a problem deserving in-depth study. Double-stream convolution neural network improves the practical value and technical complexity of dance motion automatic generation technology in art and cultural heritage protection, dance teaching, dance video retrieval, and dance arrangement.

## 1. Introduction

The core problem of the automatic generation system of specific dance movements is to explore the relationship between music and movements [1, 2]. People have such expectations for the music-driven dance generation effect: in the process of music playing, with the change of music, the specific dance movements will also change accordingly [3, 4]. Because people are sensitive to changes in music and human movement, they can detect some subtle changes. For example, the same music rhythm can express different emotions, and the same movement can show different dance styles. Dance-specific movement recognition can also obtain and save the key information of dance movements, so as to reduce the risk of disappearance of dance in the process of inheritance. Data collection and preprocessing, dance feature extraction and construction, and dance action recognition are currently the three steps that make up the main dance-specific action recognition process [5, 6]. The core of dance gesture recognition is the extraction and construction of dance features, but existing feature extraction and construction techniques, such as those based on simple feature tracking and meaning, frequently lack accuracy.

RETRACTED

The accuracy of dance-specific movement recognition is somewhat improved by the fault-tolerant feature expansion of standard sign language recognition under the condition of limited samples, but there is still the problem that the recognition accuracy is not high. It is necessary to combine the key information of particular dance movements in order to solve this issue. A dual-stream convolution neural network is suggested in this paper to investigate the recognition of particular dance movements. Two streams make up the two-stream convolutional neural network (CNN) [7–9]. One video frame is used as the input for the spatial stream, which is in charge of extracting background and object information from the video. For instance, spatial flow can be used to identify the two essential details of the man and ball's appearance in ball games. The two-stream convolution neural network uses its input data independently for the space stream and time stream to recognize behavior. A softmax prediction score will be assigned to each stream. The prediction scores of the two streams are combined to produce the final discrimination result. Typically, optical flow is used to represent the timing or motion of video. The main reason optical flow is so effective in behavior recognition models is that it is independent of how an image looks. As a result, optical flow is used as the model input for the time flow convolution network. The optical flow displacement field is also stacked between several consecutive frames to create the model's input. Because the network does not need to implicitly estimate the motion, this operation strengthens the motion trend and characteristics in the optical flow, allowing the model to obtain a better recognition effect [1, 10].

With the aid of specialized software and hardware, dance-specific motion recognition captures human motion behavior, and the task of motion data representation is to express the captured motion information as a data structure that the machine can understand for the purposes of analyzing and recognizing various types of motion data later [11]. The optical flow image used as the input for the dual-stream convolution neural network was created by superimposing the optical flow data from several consecutive video frames. It can effectively extract the time information from the motion video, reflect motion information between frames with clarity, and increase the precision of motion recognition. The network's next layer neuron receives its input from the previous layer neuron node's output. The network model can automatically learn more complex features through the operation of pooling layers and the training of multiple convolution layers [12, 13]. The double-stream convolution neural network enhances the practical value of the automatic dance motion generation technology in the preservation of artistic and cultural heritage, dance instruction, dance video retrieval, and dance arrangement, as well as the technology's complexity, which has grown to be a concern deserving in-depth research [14]. It makes it possible to identify particular dance moves in intricate dance scenes. It has been demonstrated through an experiment with a double-stream convolution neural network that this technique can successfully extract the specific motion feature data of human dance and enhance the precision of dance-specific motion recognition. In this paper, the following two innovations are put forward, and the contents are as follows.

1. In this paper, a double-stream CNN model diagram is constructed. Two groups of networks, spatial flow and time flow, are designed by the dual-stream CNN model. They are trained on the single video frame and the optical flow images extracted from consecutive frames and extract the spatial information and time information of the motion. The input image of spatial network is a single-frame video image, and the human motion information in the video frame can be identified by feature extraction of the static video frame. In a sense, the static image frame is very valuable for distinguishing the motion information. The input of time stream is the stacked optical flow graph between consecutive video frames, and the displacement of objects in the scene between two consecutive frames due to motion is called optical flow.
2. The effectiveness of the dance recognition algorithm is examined. The position of human joints is determined using a double-stream convolution neural network algorithm, and the dance instructors' posture is determined based on the angle and posture of their fixed axis joints. A database of typical dance movements is then established as a benchmark for dance training.

RETRACTED

## 2. Related Work

Dance-specific movements have high complexity, and dance movements also have many problems such as self-occlusion. The research on motion recognition based on dance video needs to be further developed. Many scholars have carried out research on a large number of dance-specific movements.

Liu et al. regarded human posture estimation as a detection problem and estimated human posture by regression of the thermal map of key points of human posture. After that, a human posture estimation method using the response diagram of human components to express the spatial constraints between components was proposed [2]. Nguyen et al. proposed that the dance movement can be regarded as a continuous set of postures, so it needs to be represented by the information of multiple images. In order to extract human motion features from the preprocessed images, not only should the feature information in the image at a certain time be extracted, but also the correlation between the motion features of adjacent images should be established [15]. Thomas et al. state that the purpose of human dance-specific action recognition is to analyze and understand human body actions and behaviors in video. Different from object recognition in two-dimensional space in static images, behavior recognition mainly studies how to perceive the spatiotemporal motion changes of target objects in image sequences and expands the expression form of human dance-specific actions from two-dimensional space to three-dimensional space [16]. Zheng et al. can identify and track the targets in the dynamic scene by analyzing the dance-specific action image sequence of the video. On this basis, the target behavior is analyzed to facilitate immediate response in case of emergencies [17]. Krishna proposed a human posture estimation algorithm based on hourglass, which can obtain multi-scale features and have a more concise structure [18]. Sun pointed out that music rhythm plays an important role in Latin dance and good music accuracy is the basis for high-level players to achieve excellent results. The practice of music rhythm and Latin dance, through the analysis of the music form in the competition, discusses the processing method of music rhythm and summarizes the impact of music processing on Latin dance competition so that Latin dancers can more clearly understand the importance of music processing to the competition, master more reasonable music processing methods, provide reference for future training and competition, and promote the improvement of their performance [19]. The interactive learning method was provided by Sun et al. in view of the current music rhythm problems such as students' weak sense of music, outdated teaching methods, and poor coordination between dance movements and music rhythm. This paper suggests that music rhythm teaching in sports dance should pay attention to cultivating students' music literacy, improving teaching methods, and strengthening the organic coordination between dance movements and music festivals. Only by paying attention to the teaching of music rhythm can we effectively improve the performance level of specific dance movements [20]. According to Zhou et al., the main principle of the method of real-time detection of multi-person 2D posture is to learn to associate body parts with corresponding individuals through partial affinity domain [21]. Stange also reflects the misidentification of specific movements of each dance, which can provide guidance for improving the parameters of classification feature extraction [22]. Wang et al. believe that the research results of specific motion recognition technology of dance video not only help dance professionals analyze dance video, but also can be used for teaching, protecting, and mining artistic and cultural heritage [23].

RETRACTED

In this study, the recognition of particular complex dance movements is learned using a two-stream convolution neural network algorithm. The human body region is identified by residual network based on the contour value of human key points. The classification of particular dance movements can finally be realized through the integration of key point feature classification and image classification. To ensure the accuracy of training and enhance the interactivity of dance learning, the double-stream convolution neural network algorithm is used to recognize and collect dance movements.

## 3. Dance-Specific Action Recognition Based on Double-Stream CNN

### 3.1. CNN

CNN is a new technique that typically produces good results in many tasks, including speech recognition and visual image analysis. The first use of CNN, a specially created deep model, was in the area of image recognition [24, 25]. Local receptive field, weight sharing, and spatial downsampling—which greatly reduce the number of weight parameters in the network and achieve invariance to image displacement, scale, and deformation—are the fundamental concepts of CNN. To reduce the dimension of convolution features and produce space-invariant features, sampling operations calculate the average or maximum value of all pixels in the sampling range as the sampled value of the region. The maximum downsampling operation is used in this paper. Because the cells in the visual layer of the biological brain are more inclined to perceive the stimulation of local areas, it does not follow biological principle to fully connect all the pixels in the input image with each neuron in the next layer. The biological process of perceiving things involves moving from the small to the big picture. The small details are controlled first, and then macro cognition of the entire system is created. The architecture of CNN is shown in Figure 1.

The convolution layer is made up of a number of parallel characteristic graphs that are created by sliding various convolution kernels over the input image and applying particular operations to them. Additionally, the convolution kernel and the input image carry out an element-by-element multiplication and summation operation at each sliding position to project the data in the receptive field onto the functional graph's elements. The formula below can be used to determine the size of the convolution layer:

(1) $$\begin{array}{c} \text{Dim}\left(H,W,D\right)=\left(H+2Z-k\right), \end{array}$$

where *H*, *W*, and *D* are the height, width, and depth of a feature map, respectively, and *Z* is zero filling.

RETRACTED

At present, the most common pooling method is simple maximum pooling. In some cases, we also use average pooling and *L*_2_ norm pooling. When the number of convolution kernels *D*_*n*_ and the step size *Z*_*s*_ are used to perform pooling operations, their dimensions can be calculated by the following formula:

(2) $$\begin{array}{c} \text{Dim}\left(H_{2},W_{2},D_{2}\right)=\left(\frac{H_{1}-k}{Z_{s}+1}\right). \end{array}$$

If the output vector of all possible outputs is *y*_*i*_=(0,1) and the event *x* with a set of input variables is *x*=(*x*_1_, *x*_2_, *x*_*t*_), the mapping from *x* to *y*_*i*_ is as follows:

(3) $$\begin{array}{c} L\left(\hat{y},y_{i}\right)=\frac{1}{t}\sum_{i=1}^{i=t}, \end{array}$$

where $L\left(\hat{y},y_{i}\right)$ is the loss function.

If $\overset{\wedge }{y}$ is the output value of *t* training samples and *y*_*i*_ is the corresponding tag value, then the mean square error is as shown in the following formula:

(4) $$\begin{array}{c} L\left(\hat{y},y_{i}\right)=\frac{1}{t}{\sum_{i=1}^{i=t}\left(y_{i}-\overset{\wedge }{y}\right)}^{2}. \end{array}$$

Allowing neurons in the same layer to share the weight of the receptive field enables them to extract the same features in various locations throughout the image because the weight corresponding to a receptive field is a feature extractor. The weight-sharing approach can concurrently significantly lower the number of network parameters. Because CNN uses a local receptive field and a weight-sharing strategy, it differs from feedforward neural networks in how it processes data of the image type.

### 3.2. Two-Stream Convolution Neural Network

It makes sense to divide a video into two components: space and time, given the structural differences between video and image data. Spatial stream and temporal stream are the two types of networks that CNN designs. To extract the spatial and temporal details of motion, they are trained using optical stream images that are taken from discrete and continuous video frames, respectively. The input of the following layer neuron in the network is taken from the output of the layer neuron before it. The network model can automatically learn more complex features through the training of multiple convolution layers and the use of the pooling layer. To obtain the training results of the spatial stream network, the single-frame RGB image extracted from the dance-specific movement is fed into the spatial stream convolution neural network [26]. The input image for the spatial stream network is a video image in one frame. By taking the characteristics of the static video frame and extracting them, the human motion information in the video frame is identified. In a sense, it is very helpful to be able to distinguish between the motion information and the static image frame. Motion recognition from still images is successfully accomplished by the spatial stream convolution neural network, which can operate on each individual video frame. Because some actions are closely linked to particular objects, the static appearance is already a helpful cue.

RETRACTED

Due to the fact that the spatial stream convolution network layer only accepts images as input and is solely a classification network, it can be studied using the most recent advancements in large-scale image recognition techniques. It has many data sets for pretraining, which is useful for addressing the issue of overfitting. A stacked optical flow graph between successive video frames serves as the input for time flow. Optical flow describes how motion causes objects in a scene to move between two successive frames. To get the time flow network's training results, the optical flow data must first be extracted from either a single frame or a series of frames before being used as the time flow network's input. The prediction scores from the two streams are then combined to produce the final discrimination result. The motion or timing information of a video is typically represented by optical flow. Because it is independent of how an image looks, optical flow is particularly effective in behavior recognition models. As a result, optical flow is used as the model input by the time flow convolution network in order to achieve the goal of time and space complementarity. A two-dimensional vector field is the basis of optical flow. Between any two consecutive frames, each vector corresponds to the point's displacement. It can be used to represent object motion because it contains data on how objects move between adjacent frames. The model diagram of double-stream convolution neural network is shown in Figure 2.

CNN dual-stream: the core of this model lies in the “double-stream” structure composed of space-stream CNN and time-stream CNN. A deeper hierarchical structure, fewer filters, a smaller convolution operation step, and a smaller convolution kernel size are current trends in network structure development. Object detection has benefited from these modifications and seen positive outcomes. In comparison to AlexNet, the original dual-stream convolution neural network has more convolution filters, a smaller first convolution layer convolution kernel (66), and a smaller convolution step size (2). Other layers' parameters are the same as AlexNet [27].

RETRACTED

The input of time-stream network is processed in the following two ways: *w* and *h* represent the width and height of a video. The input *I*_*τ*_ ∈ *R* of a convolution network is set to any frame (*t*) as follows:

(5) $$\begin{array}{c} I_{\tau }={\text{d}}_{\tau +k-1}^{x}\left(u+v\right),\\ I_{\tau }={\text{d}}_{\tau +k-1}^{y}\left(u,v\right). \end{array}$$

For any point (*u*, *v*), the channel encodes all points of the *L* sequence frame.

In this case, *I*_*τ*_ is the input vector, and the following formula is used to correspond to a frame *t*:

(6) $$\begin{array}{c} I_{\tau }\left(u,v,2k-1\right)=\left(P_{k}\right),\\ I_{\tau }\left(u,v,2k\right)=\left(P_{k}\right)\text{,} \end{array}$$

where *P*_*k*_ is the *K* layer along the track. From (*u*, *v*), the following recursive relationship definitions exist between frames:

(7) $$\begin{array}{c} P_{1}=\left(u,v\right),\\ P_{k}=P_{k-1},k>1. \end{array}$$

In time flow network training, 224 × 224 × 2L frame input is randomly cropped and flipped. The learning rate is initially set at 10–2 and then reduced according to a fixed schedule. The rate of learning is constant across all training sets. The motion or timing information of a video is typically represented by optical flow. Because it is independent of how an image looks, optical flow is particularly effective in behavior recognition models. In order to use optical flow as a model input, the time flow convolution network does so. The optical flow displacement field is also stacked between a number of successive frames to create the input for the model. The network does not have to estimate the motion implicitly, which strengthens the motion trend and characteristics in the optical flow and improves the recognition effect of the model. Due to the fact that the spatial stream convolution network layer only accepts images as input and is solely a classification network, it can be studied using the most recent advancements in large-scale image recognition techniques. It has many data sets for pretraining in order to address the issue of overfitting [28]. Once the scores of the sampled frames and video frames have been averaged, the scores for the entire video are obtained. The idea behind choosing the position of the fusion of time flow and space flow networks is to fuse the two CNNs at the same relative position. This can guarantee that the input size and the quantity of channels of the feature Tao are the same, which is helpful for network training and testing after fusion. Without taking into account how spatial and temporal data in a video relate to one another, the recognition results of spatial stream and temporal stream networks are combined by averaging. The best network structure will be found by conducting experimental research using a variety of fusion strategies in this paper.

RETRACTED

### 3.3. Performance Analysis of Dance Recognition Algorithm

Double-stream convolution neural network algorithm successfully predicted 15 joints of dancers, but there was a deviation in the prediction of joints of head and waist. This algorithm has some shortcomings in dealing with limb joints with large-scale changes. For example, for ball games, the two key appearance information items of man and ball can be identified through spatial flow. The space stream and time stream of the two-stream convolution neural network independently use their input data for behavior recognition. Each stream will get a softmax prediction score. At the same time, audio features contain a lot of information, which is an important auxiliary feature and can reduce the influence of self-occlusion in dance movements. The dancer's movement range is large, and the figure is seriously deformed relative to the human body, which interferes with the algorithm's return to joint points. However, the dual-stream convolution neural network algorithm can accurately predict the dancer's skeleton nodes in general, which proves that the algorithm is effective. The video data of dance-specific movements are extracted by frames to generate picture sequences, the picture sequences are used as the input of PAFs, and the posture of each picture is estimated to obtain the spatial skeleton node sequence. The dual-stream convolution neural network input image is an optical flow image generated by superimposing the optical flow information of multiple consecutive video frames. It can clearly reflect the motion information between frames, effectively extract the time information in the motion video, and help to improve the accuracy of motion recognition. Each dance action selects 5 frames from its picture sequence for display. The performance of human posture estimation algorithm directly affects the generation of spatial skeleton node sequence and then affects the recognition of dance movements.

Double-stream convolution neural network algorithm is used to identify the position of human joints, the human posture of dance trainers is identified based on the angle and posture of fixed axis joints, and the standard dance movement database is established as a comparison template for dance training. Trainers learn dance movements through the double-stream CNN algorithm, and after successfully obtaining the spatial skeleton node sequence of dance video data, they are now identified by the classifier. The spatial skeleton node sequence of dance video data corresponds to the videos in the data one by one and also contains 10 classic dance movements. Dance-specific motion recognition records human motion behavior with the help of specific software and hardware equipment, and the task of motion data representation is to express the captured motion information as a data structure acceptable to the machine for the purpose of subsequent analysis and recognition of various types of motion data. Through the training of multiple convolution layers and the operation of pool layers, the network model can automatically learn more complex features. Double-stream convolution neural network improves the practical value of automatic dance movement generation technology in the protection of artistic and cultural heritage, dance teaching, dance video retrieval, and dance arrangement. Experiments show that the double-stream convolution neural network algorithm can accurately identify the dance trainer's movements and give evaluation data, which can effectively improve the trainer's dance level.

RETRACTED

## 4. Analysis and Discussion of Simulation Results

### 4.1. Model Training and Experiment

The coordinates of each action joint point of the trainer are collected, and the difference between the actions is visually found by comparison with the motion trajectory of the joint point of the standard action. The comparison data of the joint coordinates of the two action parts are shown in Table 1.

From the experimental results, it can be seen that there is a big deviation between the coordinates of the trainer's arm and the coordinates of the standard movement joints. The height of the trainer's arm has not reached the predetermined value, the wrist needs to be increased by 152 mm, and the swing amplitude and frequency are too fast, which makes the training dance posture inconsistent with the standard movement.

At the same time, the training action information is collected to obtain the joint angle comparison as shown in Table 2.

From the experimental results, it can be seen that the angle of the right wrist, elbow, and shoulder of the trainer is larger than that of the standard movement. Therefore, during the training process, it is necessary to correct the movement, such as bending the right leg, straightening the right arm, and leaning forward.

RETRACTED

The corresponding relationship between music and dance-specific motion matching calculation is complex, and the matching characteristics contained in the corresponding relationship between different kinds of dance and music are very different. For a specific kind of dance, determining the corresponding relationship between music and action is of great significance to the implementation of music-driven dance action automatic generation system. After calculating the correlation coefficients of all music and dance-specific action characteristics, a correlation coefficient matrix is obtained. This experiment aims to test the change rate of eigenvalues of foot track and root mean square of energy in tap dance. The experimental results are shown in Figure 3.

As can be seen from Figure 3, the higher the correlation coefficient of dance-specific movement features, the higher the synchronicity of the change rates of the two feature values. With the increase of the number of training samples, the change rate of eigenvalues fluctuates greatly, and the footstep track changes with the root mean square of energy.

In order to further verify the recognition efficiency of this algorithm, tests are carried out in scenes with 0 to more than one person, and the efficiency experimental results of different people are shown in Figure 4. The algorithms in literature [1] and literature [2] and the algorithm in this paper are used to test the efficiency. The efficiency of different numbers of people is shown in Figure 4. The efficiency under different algorithms is shown in Figure 5.

Figures 4 and 5 show that the amount of time spent by this algorithm increases gradually, albeit only slightly, with the number of people in the image. The algorithm in [1] and the algorithm in [2] both have linearly increasing running times as the population grows. Comparatively speaking, the running time of the algorithm in this study has not really changed all that much. As a result, this algorithm performs better and is more efficient.

### 4.2. Results and Analysis

The data set of dance-specific actions used in the experiment contains 13,324 dance-specific action videos, with an average of 184 clip video frames per video. If every extracted image is sent to neural network for training and learning, the workload will be huge and there will be a lot of redundant information. The effects of video sampling frames on spatial stream and temporal stream CNN are compared experimentally, and the experimental results are shown in Table 3.

From the experimental results, it can be seen that with the increase of the number of sampling frames, the recognition rate of spatial flow and temporal flow CNNs is on the rise. When the number of sampling frames reaches 15, the recognition rate of both spatial flow and temporal flow networks is not very obvious. When the number of sampling frames is greater than 26, the recognition rate basically remains unchanged. Therefore, setting the number of video sampling frames to 25 can not only effectively extract the action image frames covering key frames, but also reduce the workload of network training.

RETRACTED

In this experiment, the spatial flow network and the time flow network are trained independently, and the same average fusion method as the original two-stream network is adopted to observe the influence of the deepened network structure on the recognition rate. The model has been trained for 200 rounds, and the experimental results of recognition accuracy are shown in Figure 6. The experimental results of recognition error rate are shown in Figure 7.

As can be seen from Figures 6 and 7, the final average recognition accuracy of spatial flow network is 76.65%, that of time flow network is 70.05%, and the final accuracy of them is 73.35% by means of average fusion. Compared with the original two-stream network's recognition accuracy of 72.15%, the recognition performance is slightly improved. As can be seen from Figure 7, the final identification average error of spatial flow network is 0.92, the final average error of time flow network is 1.67, and the final error of both is 2.59 by means of average fusion. Compared with the 3.89 identification error of the original two-stream network, the error identification performance has been gradually improved.

## 5. Conclusion

Manual guidance is typically used in traditional dance-specific movement training, which is ineffective and hazy. Professionals must invest a lot of time in listening to and analyzing the current large volume of music and dance video data. Without a doubt, this approach is very ineffective. In this paper, a dual-stream convolution neural network is used to study the recognition of particular dance movements. The time spent by this algorithm gradually increases as the number of people in the image does, but only slightly. The algorithm in literature [1] and the algorithm in literature [2] both experience linear increases in running time as the population grows. In contrast, the running time of the algorithm in this study essentially increases negligibly. This demonstrates that this algorithm is more effective and performs better. The ability of the dual-stream convolution neural network algorithm to precisely detect and recognize the dancer's movements in the dance video images makes it extremely useful for applications such as dance video movement analysis. Despite significant advancements in the stage of human pose estimation, there are still some flaws in the human joint recognition. In the subsequent work, the dual-stream convolution neural network algorithm will be enhanced.

RETRACTED

## Figures and Tables

**Figure 1:** Structure of CNN.

**Figure 2:** Model diagram of double-stream convolution neural network.

**Figure 3:** Change rate of eigenvalues of footstep track and root mean square of energy in tap dancing.

**Figure 4:** Efficiency of different numbers of people.

**Figure 5:** Efficiency under different algorithms.

**Figure 6:** Recognition accuracy of convolution neural network for spatial flow and time flow.

**Figure 7:** Identification error of convolution neural network between spatial flow and time flow.

**Table 1:** Comparison of trainer's movement and standard movement data.

Position	Training point coordinates		Standard joint point coordinates	
	Abscissa	Ordinate	Abscissa	Ordinate
Head	−69.7	269.5	−80.5	217.5
Neck	−69.7	74.6	−27.7	32.5
Left shoulder	−208.5	−3.7	−150.2	-50.5
Right shoulder	90.2	−0.8	47.4	507.7
Left knee	−25.5	−847.4	−237.6	−953.7
Right knee	−127.6	−824.5	−107.2	−862.5

**Table 2:** Comparison of joint angles.

Position	Action	
	Trainer	Standard maker
Right wrist, left elbow, left shoulder	172.4	169.5
Right wrist, left elbow, left shoulder	149.6	107.4
Waist, left knee, left ankle	158.6	153.6
Waist, right knee, right ankle	158.7	152.7

**Table 3:** Influence of the number of video sampling frames on the model recognition rate.

Frame number	Accuracy of spatial flow network identification	Accuracy of time flow network identification
15	82.22	74.02
10	84.14	74.57
15	84.56	74.72
25	84.62	75.14

## Data Availability

The data used to support the findings of this study are available from the author upon request.
